# Simulation Study on Complex Systems of Forest Biomass Power Generation Supply Chain in China

**DOI:** 10.1155/2022/7202352

**Published:** 2022-03-29

**Authors:** Ning Ma, Zhao Huang, Yue Qi

**Affiliations:** School of Economics & Management, Beijing Forestry University, Beijing 100083, China

## Abstract

Based on the perspective of complex system management of forest biomass power generation (FBPG) supply chain, this paper explores a new way to reduce the operation cost of forest biomass raw materials supply chain and improve the operation efficiency of forest biomass supply chain in China. Firstly, the supply chain model of FBPG is summarized through the survey data, and the existing problems are found. Then, the behavior strategies among farmers, middlemen, and enterprises are analyzed, and the data that cannot be obtained in the model are estimated by using statistical methods. Finally, the complex supply chain system is simulated by computer. Through setting different forestry policies, this paper compares and analyzes the profit of the supply chain and puts forward policy suggestions to promote the development of the FBPG industry in China. In this paper, the actual situation, principles of statistics, and system simulation are effectively combined to make the behavior rules of various stakeholders fit the reality, and the research conclusions are more practical.

## 1. Introduction

With the development of society, the importance of the ecological environment has become increasingly prominent. As a renewable and clean energy industry, biomass energy industry is of great significance to improve environmental quality and develop circular economy. Forest biomass power generation (FBPG) industry is an important part of biomass energy industry. It can generate economic benefits by making rational use of forestry resources and bring substantial ecological benefits by reducing pollutant emissions to protect the natural environment. Especially for the northwest area with poor natural conditions in China, the energy development of tending residues such as pruning shrubs can improve the income level of local farmers and the local natural environment.

Although the utilization of forest biomass energy is essential, China's FBPG industry is still in the initial stage of development, and there are many problems in actual development. For example, farmers lack the will to collect, so it is difficult to collect forest biomass raw materials on a large scale. In addition, the cost of raw materials remains high, and the degree of marketization is low. Therefore, from the perspective of the complex system of forest biomass raw materials supply chain, it is of great significance to mobilize the enthusiasm of farmers to collect and reduce the cost of raw materials by optimizing the policy combination so as to maximize the overall profit of the supply chain and ensure the sustainable and stable operation of biomass power generation enterprises.

This paper combines the supply chain of FBPG with computer simulation technology. Firstly, the paper models the complex supply chain system composed of farmers, middlemen, and biomass power generation enterprises and constructs a multiagent raw materials supply chain simulation model. Then, the paper puts forward the optimal combination scheme and policy suggestions for the development of the FBPG industry through simulating the simulation results under different parameters, which has important practical significance for expanding the scale of the FBPG industry in China.

## 2. Literature Review

Forest biomass refers to the organic matter formed by photosynthesis of woody plants such as forest trees. Forest biomass energy is the energy stored in forest biomass after conversion; that is, the energy can be used for power generation or heating through direct combustion or modern conversion technologies [1, 2]. Forest biomass resources can be divided into three categories: forest tending and pruning residues, “three forestry residues” (cutting residues, material residues, and processing residues), and energy forest mining residues. The overall availability of forest biomass energy resources in China is increasing year by year, and the supply capacity is significant. In particular, Inner Mongolia has the most extensive available forest biomass energy resources, accounting for 9% of China [3]. The forest biomass energy industry in the western region has great development potential.

The development of the biomass energy industry still faces problems such as difficult raw materials collection, low equipment utilization, and high operation and maintenance costs [4, 5]. By 2016, the global consumption of biomass power generation accounted for about 40% of the total consumption of biomass energy [6]. Energy has not been fully utilized, which restricts the sustainable development of biomass energy industry to a great extent. Insufficient purchase of raw materials is one of the important factors limiting the development of forest biomass energy industry [7]. At present, China's forest biomass energy mainly depends on government policy support [8]. It is urgent to explore the enthusiasm of various agents from the internal system and put forward corresponding incentive measures.

The simulation modeling method based on multiagent started in the late 1990s. This method adopts bottom-up modeling thought and emphasizes the authenticity of microindividuals during modeling. The model establishes the relationship between agents through the message mechanism and then forms the macroframework of the simulation system. Many scholars have applied multiagent simulation technology to the supply chain of forestry, agricultural products, and other fields. For example, Hanafizadeh and Sherkat [9] built a supply chain distribution model based on multiagent system, improved the convergence of agent adaptability by introducing a genetic algorithm, and then studied the related problems of distribution in supply chain management. Wang et al. [10] used NetLogo software to build a simulation model of agricultural product supply chain and explored the relationship between supervision, farmers' cooperation, and agricultural product quality. Zhang and Lin [11] established a simulation model based on multiagent to study the impact of the subsidy policy issued by the Chinese government on the profit distribution of supply chain members and carried out experiments under different subsidy levels. Terrada and Ouajji [12] applied multiagent simulation technology to the complex system of supply chain management to provide solutions to the decision-making problems among supply chain members. Awaga et al. [13] built a simulation analysis model of enterprise green product production behavior with multiagent participation and simulated the impact of different government guidance and supervision strategies on the strategic choices of two parties (enterprises and government). In addition, few scholars have studied biomass power generation industry. Shastri et al. [14] simulated biomass supply system in Illinois based on multiagent simulation technology, and the simulation revealed the impact of miscanthus energy crop on raw materials supply contract. Li [15] established an industrial system model including farmer, enterprise, market, and government and put forward suggestions on the construction scale of China's straw power generation and the centralized utilization of straw. Luo [16] constructed four biomass raw materials supply game models based on game theory and multiagent simulation technology. Then he analyzed the effect, applicability, and corresponding implementation strategies of biomass power generation raw materials supply mode.

Because of the different characteristics of supply chains, there are also differences in agent behavior rules. The multiagent modeling of the FBPG supply chain is more considered from the perspective of raw materials supply. According to the research results, farmers, middlemen, and enterprises can be abstracted as agents with independent decision-making, learning, and memory ability. There are obvious differences in the decision-making rules of agents, the interaction rules between agents and between agents, and the external environment. The use of multiagent simulation technology shows obvious advantages. The behavior rules of simulation agents are designed according to the actual behavior of individuals. Through the interaction of microagents, various emergent behaviors and self-organization phenomena in the system can be effectively explored [17].

In conclusion, the forest biomass energy industry has extensive development space. The existing problems are mainly backward technology, lagging policy, insufficient supply of raw materials, and high production cost. Therefore, it is necessary to study the supply chain of forest biomass energy raw materials from the perspective of microagents. Policy factor greatly impacts biomass power generation industry, which can promote industrial development through economic policy adjustment. In addition, although the multiagent simulation method is not widely used in the forest biomass energy supply chain, there have been many studies in the field of forestry and agriculture. Therefore, it is reasonable to summarize the industrial policy suggestions through a series of simulation experiments.

## 3. Forest Biomass Power Generation Supply Chain

### 3.1. Characteristics of Supply Chain

The characteristics of FBPG supply chain are as follows:

1. As a biomass enterprise, the power generation product cannot be saved.
2. Raw materials have a wide production area and large output, but the collection has periodicity and is greatly affected by factors such as environment and season.
3. There are many alternative uses of raw materials, resulting in large supply fluctuation.
4. Raw materials are susceptible to moisture and decay, with low weight and value density. The cost of transportation and storage is high.
5. The raw materials supply of enterprise is generally subject to many farmers and middlemen. The enterprise does not occupy a dominant position.

It can be seen that FBPG supply chain is essentially different from the conventional production supply chain. The latter usually only focuses on the uncertainty of the consumption market, while the former pays more attention to the uncertainty of upstream raw materials supply.

In addition, compared with biomass raw materials such as straw, the geographical distribution of forest biomass raw materials is more special, the collection quantity is more uncertain, and the transportation cost is more expensive. Therefore, the upstream of FBPG supply chain is relatively complex, and the supply is unstable. By signing contracts and expanding the scope of purchase, the cooperative relationship between various agents can be stabilized. When establishing the simulation model, seasonal and other random factors will be set to reflect supply uncertainty.

### 3.2. Composition of Supply Chain

The first-hand data used in this paper was obtained by issuing questionnaires in Wushen Banner and Hangjin Banner of Inner Mongolia Autonomous Region, and Zhongwei City of Ningxia Hui Autonomous Region, as well as in-depth interviews with enterprises' leaders. The survey covers the basic information and raw materials purchase information of enterprises. In this survey, 5 enterprises were visited, and 127 questionnaires of farmers related to biomass energy were completed. Fifty-four farmers have sold raw materials in two ways (Table 1).

In the upstream supply chain of FBPG, there are mainly two kinds of raw materials transportation modes. One is that forest farmers directly sell to FBPG enterprises; the other is that forest farmers sell to middlemen and then sell to enterprises by middlemen. The downstream supply chain is relatively simple. The only customer is the State Grid Corporation of China (SGCC). The whole FBPG supply chain system can be shown in Figure 1. Next, the supply chain is divided into cost supply chain and sale supply chain to analyze the upstream and downstream customers outside the enterprise.

#### 3.2.1. The Upstream Supply Chain

The upstream supply chain of FBPG enterprises in China is mainly two-level or three-level supply chain: (1) two-level supply chain: farmers/upstream companies/enterprises (independently cultivated raw materials)-power generation enterprises; (2) three-level supply chain: farmers-middlemen-power generation enterprises. Specifically, power generation enterprises mainly obtain raw materials through four modes: first, power generation enterprises independently cultivate economic forests as raw materials for power generation; second, enterprises cooperate with upstream companies to obtain raw materials, which are generally molding fuel enterprises; third, enterprises purchase crops or forest residues from farmers; fourth, enterprises purchase raw materials from middlemen. These middlemen are mainly individual farmers. Due to the market economy, they have spontaneously become a hub connecting upstream and downstream raw materials.

The choice of raw materials supply mode depends on many factors such as business plan, capital status, geographical location, and other factors. Enterprises often choose mixed modes. Mode 1 belongs to internal production of enterprises and has a low degree of application. Mode 2 is interest cooperation among enterprises. Mode 3 and mode 4 are transactions between individual farmers and enterprises. Therefore, this paper mainly studies mode 3 and mode 4.

#### 3.2.2. The Downstream Supply Chain

The downstream supply chain of FBPG is a two-level supply chain: power generation enterprises-SGCC. In addition to a few enterprises using the advantage of biomass power generation to increase sideline income, SGCC is the only downstream customer in the sale chain of the whole industry. Therefore, the formulation of policies on FBPG largely determines the survival and development of power generation enterprises.

At present, the feed-in tariff standard of biomass energy in China is 0.75 yuan/kWh. The feed-in tariff is the price of power commodity delivered to SGCC by power production enterprises. As China has formulated the priority scheduling policy, the sale of biomass power generation will be guaranteed. Moreover, according to the Renewable Energy Law, biomass power is preferentially connected to the grid and does not participate in peak regulation. Therefore, these policies reduce the impact of changes in electricity consumption of end customers on biomass power generation industry and ensure the stability of sale of biomass power generation enterprises.

## 4. Construction of the Simulation Model

This part establishes the three-level supply chain simulation model consisting of farmers, middlemen, and biomass power generation enterprises and uses NetLogo software for simulation. The role of the government appears in the form of subsidy parameters in the simulation system. The behaviors of farmers and middlemen adopt the “economic man” hypothesis. Middlemen will adjust their purchase scope according to the price of enterprise to maximize their profit. The simulation system takes enterprise as the core node of the whole supply chain to simulate the optimal purchase price and government subsidy when the enterprise reaches production capacity. The parameters and some processes of the model are mainly based on the relevant data of the Maowusu biomass thermal power plant in Erdos, Inner Mongolia. The enterprise takes the branches of sandy shrubs (mainly *Salix psammophila*) pruned from the roots as raw materials.

### 4.1. Simulation Assumptions and Process

Under the premise of ensuring the authenticity of the system as much as possible, the simulation model is simplified, and the following assumptions are made according to the actual situation:

1. There is only one biomass power generation enterprise in a particular region, and there is no competition for raw materials among multiple biomass power generation enterprises.
2. During the simulation period, the area of woodland and the number of labor forces in the region do not change, and the positions of biomass power generation enterprise, middlemen, and farmers do not change.
3. The enterprise has no difficulty in selling products; that is, all electricity can be sold, and the enterprise is only responsible for purchase, not transportation.
4. According to the current policy, the government implements the tax policy of “immediate levying and refunding,” so the impact of bank tax is not considered in the model.
5. Farmers know the purchase price of middlemen and enterprise last time before pruning. The behaviors of farmers adopt the “economic man” hypothesis.
6. The distribution of forest biomass resources is extensive, uniform, and unitary. The woodland area is infinite. The species are single, and all of them are *Salix psammophila*. They are evenly distributed in the region.
7. Middlemen take the initiative to purchase raw materials from farmers' homes.

In the simulation processes of FBPG supply chain, firstly, initialize the system state to generate the farmer agent, the middleman agent, and the biomass power generation enterprise agent. Secondly, the enterprise sets the price for purchasing raw materials, and middlemen set a reasonable purchase range according to the current price. Thirdly, farmers decide whether to collect and sell forest biomass raw materials according to the purchase price of enterprise and middlemen. If the farmers sell to middlemen, the middlemen are responsible for transportation and primary processing and then sell to the enterprise; if farmers sell directly to the enterprise, farmers need to pay the cost of transportation. After purchasing raw materials, the enterprise processes and generates electricity and then sells electricity to SGCC to obtain government subsidy. Finally, calculate the profit of the biomass power generation enterprise. Judge whether the quantity of purchase can meet the demand of enterprise. If the enterprise reaches the production capacity, the program will stop; if the production capacity is not reached, the enterprise will increase the purchase price until the program stops when the production capacity is reached. At the same time, calculate the profit of farmers and middlemen in each cycle.

The simulation system finally solves the following three problems: (1) How much purchase price can make the biomass power generation enterprise reach production capacity and obtain the maximum ecological benefits. (2) How much government subsidy can ensure that the enterprise does not lose money at the purchase price of reaching production capacity. (3) What policy can be implemented to improve the overall efficiency of the supply chain.

### 4.2. Construction of the Simulation Model

#### 4.2.1. Property and Parameter Setting of the Farmer Agent

According to the survey data of Inner Mongolia, about 140 farmers directly transport raw materials to the enterprise every year, involving 100–300 kilometers. About 20 middlemen transport raw materials to the enterprise every year, also involving 100–300 kilometers. Each middleman purchases raw materials from about 20 farmers. Therefore, there are about 540 farmers involved in selling raw materials. At the same time, in the farmers' questionnaires, the number of farmers who have sold raw materials in recent three years accounts for 48.1% of the respondents. It is roughly estimated that the number of forest farmers within 300 kilometers of the enterprise is about 1123. Moreover, because farmers prune every three years, it is estimated that the number of farmers is about 3369. Each 1/15 hm^2^*Salix psammophila* can produce about 1t branches [18]. However, pruning *Salix psammophila* is greatly affected by external factors such as season and family labor force. The actual unit collection is often less than 1t. Therefore, a random variable *α* (value between 0.5∼1) is designed to more truly reflect the pruning situation of farmers. The pruning cost is mainly labor cost, and the pruning cost per ton of raw materials is about 70∼200 yuan.

According to the survey, the woodland area of farmers ranges from 5 to 5400 mu. Through the K-S test, the woodland area data is not a normal distribution, and there are obvious abnormal values. Clean the woodland area data, sort the data from small to big, and take 25% as the upper quartile FL and 75% as the lower quartile Fu. The quartile distance IQR is Fu-FL. Then the upper bound of the data is *Fu*+1.5 × IQR, the lower bound is FL − 1.5 × IQR, and the data ranges from 5 to 1585 mu after cleaning.

Grouping the data with 200 as group interval, it can be found that the data distribution is close to the exponential distribution. After fitting the exponential distribution, the fitting function and goodness of fit are obtained, and the fitting effect is good, as shown in Figure 2.

Based on the previous analysis and survey data, the main parameters of the farmer are sorted into Table 2.

#### 4.2.2. Property and Parameter Setting of the Middleman Agent

Middlemen purchase branches from farmers but are not responsible for the harvesting and collecting branches. The purchase price is 180 yuan/ton. The cost of raw materials primary processing (including chipping and bundling) ranges from 20 yuan/ton to 35 yuan/ton. The main parameters of the middleman are sorted into Table 3.

#### 4.2.3. Property and Parameter Setting of the Enterprise Agent

1. Calculation of raw materials demand of the enterprise: taking Maowusu power plant as an example, the unit installed capacity is 2 × 12 MW, and the power generation per hour is 2 × 1.2 kW. As pruning and collecting of *Salix psammophila* occur on the sand, the raw materials after chipping contain a large amount of sand. It is necessary to shut down for 20–25 days every year to clean the tube wall; otherwise, the pipeline will be blocked and the service life of the unit will be reduced. Therefore, if the generator unit reaches production capacity, assuming that it needs to be shut down for 25 days, the annual power generation is 195.84 million (2 × 1.2 × 24 × 340) kWh. According to the survey data, 1.25 Kg *Salix psammophila* can be converted into 1 kWh, so at least 156672 tons (19584 × 10^4^/1.25/10^3^) *Salix psammophila* can meet the needs of the enterprise. In fact, considering that the enterprise has other raw materials besides *Salix psammophila*, the demand is about 100000 tons. (2) Cost and profit: at present, the feed-in tariff of SGCC is 0.75 yuan/kWh, of which 0.277 is the benchmark price. Without considering the bank cost, the power generation cost per kWh is 0.292 yuan. The main parameters of the enterprise are sorted into Table 4.

#### 4.2.4. Behavior Rules of the Farmer Agent

Farmers aim to maximize their profit and choose a reasonable sale object. Farmers' profit is sale income plus government subsidy and minus all costs. Farmers need to pay the collection cost of collecting biomass raw materials; the income of farmers mainly comes from biomass raw materials in their woodland. If it is sold directly to the enterprise, it also needs to pay the transportation cost. The main influencing factors of biomass raw materials transportation cost include vehicle technical performance, vehicle operating cost, characteristics of crops, collection mode, and radius [19]. Because the actual route is generally curved, the road tortuosity factor $\lambda \left(\lambda =\sqrt{2}\right)$ is introduced for correction. At the same time, the round-trip transportation is considered, so the distance should be twice the actual distance. Therefore, some formulas of farmers' behaviors are as follows:

(1) Quantity of raw materials collected (*Q*)=FS × UAmo × *α*.
(2) Pruning cost (FC_1_)=FCost × *Q*.
(3) Transportation cost of the farmer ${\text{FC}}_{2}=2\sqrt{2}\times \text{FEd}\times$ transportation cost per unit distance.
(4) The transportation cost per unit distance varies with the collection quantity. According to the questionnaires, the type and performance of vehicles mainly used by farmers are shown in Table 5.
It is known that the average oil price in Inner Mongolia is 5 yuan/L. The transportation cost per unit distance of farmer with different collection quantity can be expressed as follows:
When 0 < *Q* ≤ 0.5, the tricycle is used for transportation, and the transportation cost per kilometer is 0.5 yuan.
When 0.5 < *Q* ≤ 1.5, the tractor is used for transportation, and the transportation cost per kilometer is 0.75 yuan.
When *Q* ≥ 1.5, the four-wheel vehicle is used for transportation, and the transportation cost per kilometer is [*Q*/2.5] yuan.
[*Q*/2.5] means to take the smallest integer larger than itself.
Therefore, the transportation cost of the farmer (FC_2_) can be calculated.
(5) The profit of farmer from selling raw materials to the enterprise is
  (1) $$\begin{array}{c} W_{1}=\text{EPri}\times \text{Q}+\text{FS}\times \text{CSub}-{\text{FC}}_{1}-{\text{FC}}_{2}. \end{array}$$
(6) The profit of farmer from selling raw materials to the middleman is
  (2) $$\begin{array}{c} W_{2}=\text{MPri}\times \text{Q}+\text{FS}\times \text{CSub}-{\text{FC}}_{1}. \end{array}$$
(7) The farmer compares *W*_1_ and *W*_2_ to choose to prune or not, and whether to sell to the middleman or sell to enterprise. Calculate the quantity of raw materials actually transported to the enterprise (*Q*_*fe*_) and the quantity of raw materials actually transported to the middleman (*Q*_*fm*_) in each cycle.

The specific behavior rules of farmer are shown in Figure 3.

It should be noticed that *Salix psammophila* matures in about three years, and the more it is cut, the more lusher it is. If the grown branches are not cut off, it will become dead branches in less than seven years. Because the government has public welfare forest subsidy for energy forest, once *Salix psammophila* dies, farmers will not be able to obtain public welfare forest subsidy, which will cause great losses to farmers. Therefore, the system assumes that farmers must choose to prune in the cycle, and the frequency of pruning is set to one time every three years. Moreover, the purchase scope of the middleman may not cover all farmers, so the farmer needs to judge whether he/she is within the purchase scope of the nearest middleman in advance so as to make the next decision of choosing to prune or not and selecting sale object.

#### 4.2.5. Behavior Rules of Middleman Agent

Middlemen also aim to maximize their profit and hope to acquire and sell as many raw materials as possible. Middlemen are responsible for the initial processing and transportation of raw materials in the supply chain. The transportation route consists of two parts: one is that the middleman purchases from the farmer and then transports raw materials to the processing point (the location of the middleman), and the other is that the middleman transports raw materials from the processing point to the biomass power generation enterprise. Middleman decides the current purchase scope based on the current purchase price of the enterprise.

According to the questionnaires, there are two main types of vehicles used by middlemen, as shown in Table 6. It is assumed that a large four-wheel vehicle is mainly used when middleman purchases raw materials from retail farmers, and a truck is mainly used to transport the biomass raw materials after chipping to the enterprise. Because the middleman can purchase from multiple households at the same time, it can be seen that the vehicle is always fully loaded during the purchase of raw materials from retail farmers:

1. When middleman purchases raw materials from retail farmers, the unit transportation cost is 0.25 yuan/ton·km (the calculation formula is 25 × 5/100/5).
2. Because the middleman cannot accurately estimate the purchase quantity before determining the purchase scope, the unit transportation cost transported to the enterprise is temporarily calculated as full load so as to calculate the purchase radius R of the middleman.
3. The estimated unit transportation cost of transporting raw materials to the enterprise is 0.067 yuan/ton·km (the calculation formula is 40 × 5/100/30).
4. The purchase radius *R* of the middleman should base on the economy of cost. According to the calculation method of purchase radius in reference [20], the unit cost of the middleman should be less than the purchase price of the enterprise (EPri). The road tortuosity fact.or and round-trip transportation which are the same as farmers are considered. The formula is expressed: $\text{MPri}+\text{MCost}+2\sqrt{2}\times 0.25\times R+2\sqrt{2}\times 0.067\times \text{MEd}\leq \text{EPri}$

The maximum purchase radius of the middleman is

(3) $$\begin{array}{c} R=\frac{\text{EPri}-\text{MPri}-\text{Mcost}-\sqrt{2}\times 0.133\times \text{MEd}}{\sqrt{2}\times 0.5}. \end{array}$$

(1) The purchase quantity of the middleman is the sum of the quantity of raw materials within the purchase scope:
  (4) $$\begin{array}{c} Q_{m}=\sum Q_{fm}. \end{array}$$
(2) The primary processing cost of the middleman is MC_1_=MCost × *Q*_*m*_.
(3) The actual transportation cost of the middleman is
  (5) $$\begin{array}{c} {\text{MC}}_{2}=2\sqrt{2}\times \left(0.25\times \text{R}+\left[\frac{Q_{m}}{30}\right]\times 2\times \text{MEd}\right). \end{array}$$
(4) The profit of middleman is
  (6) $$\begin{array}{c} W_{3}=\left(\text{EPri}-\text{MPri}\right)\times Q_{m}-{\text{MC}}_{1}-{\text{MC}}_{2}. \end{array}$$

The specific behavior rules of middleman are shown in Figure 4.

#### 4.2.6. Behavior Rules of the Enterprise Agent

The enterprise plays a leading role in the whole supply chain. The change of enterprise's purchase price will have an impact on the purchase scope of middlemen and farmers' willingness to sell. The initial price of the enterprise is set according to the current market price. If the production capacity is not reached, the purchase price of the enterprise in the next cycle will increase by 5 yuan/ton. If output exceeds demand, the price in the next cycle will be reduced by 5 yuan/ton to reach an equilibrium state.

Some formulas are calculated as follows:

1. Price change function: EPri=EPri+5
2. Total quantity of raw materials purchased by the enterprise: *Q*_*e*_=*Q*_*m*_+*Q*_*fe*_
3. Power generation of the enterprise: *q*=800 × *Q*_*e*_
4. Power generation cost: EC_1_=0.292 × *q*
5. Purchase cost of the enterprise: EC_2_=EPri × *Q*_*e*_
6. The profit of the enterprise: *W*_4_=0.9 × Price × *q* − EC_1_ − EC_2_

In (6), 0.9 means that 90% of the electricity of the enterprise is for sale and 10% for self-use.

## 5. Analysis of Simulation Results

### 5.1. Simulation Interface and Model Verification

The initial parameters used in the simulation system come from the survey data of farmers in many towns in Inner Mongolia and Ningxia. Except for unit pruning subsidy, other parameters are assigned in the form of sliding strip. The initial values of number of farmers, number of middlemen, middlemen purchase price, and feed-in tariff are all taken from the survey data as described in Section 4.2.1. The unit pruning cost of farmers usually ranges from 70 to 200 yuan/ton, and the unit processing cost of middlemen ranges from 20 to 35 yuan/ton. The values with high frequency in the survey data are taken as the initial parameter values, which are 100 yuan/ton and 25 yuan/ton, respectively. According to the actual situation of the survey, the initial value of unit pruning subsidy is set to 10.

First, input the initial parameters into the system, as shown in Figure 5.

After inputting the initial parameters, design the view interface of the FBPG raw materials supply chain network, as shown in Figure 6 (the figure shows the transportation of raw materials in a cycle). The gray area is the woodland after pruning (*n* = 0), the light green area is the woodland within three years after pruning (*n* < 3), and the dark green area represents the woodland that can be used for pruning (3 ≤ *n* ≤ 5). Farmers are represented by small triangles, middlemen are represented by white squares, and the enterprise is represented by a red dot in the center. With the dynamic change of cycle, the interface can visually show the change of pruning and the transportation of raw materials.

Under the setting conditions in Figure 5, export the data obtained from the system to EXCEL and draw the relationship between purchase price and purchase quantity, as shown in Figure 7. According to the above analysis, the amount of raw materials required by the enterprise for power generation is about 100000 tons. If the raw materials purchased by the enterprise can meet the demand when reaching production capacity, the purchase price needs to be between 425 and 435 yuan. At this time, the purchase quantity and purchase price of the enterprise tend to be stable.

Under the setting conditions, the profit of enterprise is negative. Similarly, export the relevant data of enterprise's profit, as shown in Figure 8. After the purchase quantity and purchase price of the enterprise tend to be stable, the loss is about 1.16∼1.3 million yuan. In order to make the enterprise more profitable, government subsidy should be gradually increased; that is, the feed-in tariff should be increased.

Therefore, continue to adjust the feed-in tariff to study when enterprise generates profit. When the feed-in tariff reaches 0.85 yuan/kWh, the power generation profit of the enterprise is still negative, with a loss of about 3 million yuan. Continue to gradually increase the feed-in tariff by 0.01 yuan until 0.95 yuan/kWh, and the enterprise can achieve profitability under the condition of meeting the raw materials demand, as shown in Figure 9.

It is not difficult to find that the simulation result is basically consistent with the survey data of existing policy. At present, the purchase price of forest biomass raw materials is 400 yuan per ton, and the enterprise can only purchase 80000∼90000 tons of raw materials. In the survey, it is found that most biomass power generation enterprises are in a state of loss at the price of 0.75 yuan/kWh. Therefore, it can be verified that the model construction is basically reasonable.

### 5.2. Simulation Experiments

The previous section has verified the rationality of the model. Therefore, adjust the parameters from the perspective of supply chain, internal agent, and external environment, and further discuss the influence of parameter change on supply chain. Several comparative experiments are carried out based on the initial parameters.

#### 5.2.1. From the Perspective of Supply Chain

The policy subsidy sharing contract can help the whole supply chain achieve coordination [21]. The supply of middlemen is affected by the raw materials market. When the market supply is less than demand, middlemen need to spend a higher price to buy raw materials from other regions. It is difficult for the whole supply chain to achieve coordination in this condition. Middlemen are more inclined to seek a smaller order quantity to ensure that their profit is as large as possible. Therefore, based on the subsidy sharing contract, middlemen are willing to sign a higher order quantity with the enterprise, which improves the enthusiasm for purchase. Similarly, this kind of contract coordination is applicable to farmers and enterprises. Therefore, the enterprise can increase the overall profit of the supply chain by increasing the purchase price. How to determine the optimal subsidy proportion of the enterprise (*β*) is very important. In the above initial environment, compare the profit of middleman, enterprise, and farmer, as shown in Figure 10.

When the feed-in tariff remains unchanged (price = 0.95), two periodic nodes are selected, which are the node that does not reach equilibrium and the node that reaches equilibrium. For example, at the two nodes of *t* = 7 (not reaching equilibrium) and *t* = 17 (reaching equilibrium), the two nodes' raw materials purchase price of the enterprise is different, which are 380 yuan per ton and 420 yuan per ton, respectively. Compare the profit of each agent and the whole of the supply chain under the two nodes, and sort out the relevant data of the nodes in Table 7.

When the purchase price of the enterprise increases, the overall profit of the supply chain increases significantly, which verifies the rationality of the experiment. In this experiment, the government subsidy (*t*) is 0.673 yuan/kWh (0.95–0.277), which is equivalent to 538.5 yuan/ton of forest biomass raw materials. At this time, the purchase price is 420 yuan/ton, and the subsidy coefficient (*β*) can be calculated as 0.074.

#### 5.2.2. From the Perspective of the Internal Agent

The purchase price of enterprise plays a leading role in the whole supply chain. In addition, other parameters also have an impact on the supply of forest biomass raw materials. Such as the unit operating cost of power generation, the unit pruning cost of farmers, and the initial processing cost of middlemen. Reducing these costs can effectively improve the operation efficiency of the supply chain. Next, the paper will study which cost reduction is the most effective in improving the efficiency of forest biomass supply chain. Under the condition that the external environment parameters remain unchanged, several experiments are carried out, and the results are shown in Table 8. Because the experiments have certain randomness, the results are given according to the average level of many simulation experiments.

The unit pruning cost can continue to be reduced, and the supply chain is more sensitive to the unit pruning cost. Reducing the pruning cost by 30 yuan per mu can greatly reduce the purchase price of the enterprise. Therefore, for the western region in China, improving the mechanization level of raw materials collection and reducing labor cost will be an effective way to improve the efficiency of biomass supply chain. In addition, the reduction of the initial processing cost of middlemen did not cause great changes in the purchase price of enterprise. Because middlemen have original capital and initial investment, there is little space for the decline of unit initial processing cost. Finally, for enterprises, reducing the operation cost of power generation can effectively avoid the loss. Through technical improvement, strengthening the construction of the management team, and reducing management cost, enterprises can seek survival space under the existing feed-in tariff level.

#### 5.2.3. From the Perspective of the External Environment

Although the government is not a main agent in the forest biomass supply chain, as an important force to promote the development of the FBPG industry, policy subsidy is an important way to improve the supply of forest biomass raw materials. In addition to the feed-in tariff subsidy mentioned above, the existing subsidies include “immediate levying and refunding” for enterprise tax and pruning subsidy for farmers. In particular, the pruning subsidy of farmers is still in the exploratory stage and has important research value. In addition, it is found in the simulation that the number of farmers and middlemen in the region has a great impact on the whole supply chain. Under the condition that the internal main parameters remain unchanged, several experiments are carried out, and the results are shown in Table 9.

Pruning subsidy can effectively help reduce the purchase price of enterprise and alleviate the pressure on enterprise to purchase raw materials. The number of farmers (or woodland area) in the region has a great impact on the whole supply chain. Therefore, when selecting the site, it is necessary for enterprises to investigate the local forest biomass energy potential and choose the area with rich resources as the power generation address. The number of middlemen will also have a certain impact on the raw materials purchase of enterprises. If the number of middlemen in the region is too small, it will also increase the difficulty for enterprises to acquire raw materials. In particular, it is difficult to acquire raw materials from farmers in remote areas and small areas.

### 5.3. Result Analysis

The simulation experiment is carried out by adjusting the parameter value, and the results are summarized as follows:

1. Combined with the actual operation of the current enterprises in China, the current feed-in tariff of 0.75 yuan per kWh (including subsidy) is low for biomass power generation enterprises, and most enterprises are facing the crisis of bankruptcy. The survey also found that 69 farmers believe that the current purchase price of raw materials is unreasonable. The simulation results show that when the feed-in tariff is increased to about 0.95∼1.0 yuan per kWh, the biomass power generation enterprises will not suffer losses when reaching the production capacity. At the same time, the purchase price of the enterprises needs to be improved. Under the current purchase price, the supply of raw materials is insufficient. It is more appropriate that the purchase price of raw materials should increase about 25 yuan at the current level of 400 yuan per ton.
2. Unit pruning cost has a great impact on the whole supply chain. The increase of pruning cost will lead enterprises to reach the production capacity at a higher purchase price. At the same time, the feed-in tariff that meets the profitable conditions of enterprises will also increase. Therefore, combined with the relevant policies of energy subsidy in the western region of China, the government can adopt appropriate subsidy for purchasing agricultural machinery to realize large-scale mechanized collection and greatly reduce the cost of artificial pruning. The government gives farmers a pruning subsidy, which can also promote some farmers to participate in pruning and increase the supply of raw materials.
3. When selecting the site, biomass power generation enterprises need to take the external environment factors into account to ensure that the number of local farmers can provide enough forest biomass raw materials. In addition, the enterprises should establish a long-term and stable partnership with middlemen, reasonably plan the number of middlemen, and ensure a stable supply of raw materials.

## 6. Conclusions

FBPG industry is of great significance to protect the ecological environment and promote the increase of farmers' income in the western region of China. Research and survey found that the current bottleneck of industrial development in China is mainly due to the insufficient supply of raw materials and serious losses of enterprises. In order to solve this problem, this paper discusses the coordination of the FBPG supply chain on the premise of uncertain supply. This is a supplement to a subdivided field of straw biomass power generation supply chain research. At the same time, the combination of empirical research and case analysis makes up for the defect of excessive parameter value deviation in the simulation processes and enriches the research content of multiagent simulation of the supply chain. The conclusions of this paper are as follows.

Firstly, it is relatively difficult to collect forest biomass raw materials in China, which has a great relationship with the terrain. Farmers' collection cost is high, and they generally believe that the purchase price of enterprises is low. Because the labor income level has been increasing in recent years, this leads to the low willingness of farmers to collect and sell raw materials. In addition, forest biomass raw materials also have many other values besides being sold to enterprises, such as covering sand layer (sand-prevention) and self-use as an alternative fuel. There are many methods to sell biomass raw materials collected by farmers. The choice of farmers depends on which method can obtain the greatest profit. Therefore, through reasonably increasing the purchase price and giving subsidy for purchasing agricultural machinery, the participation of forest farmers can be improved. It is conducive to the stable supply of raw materials and helps the sustainable and stable development of enterprises.

Secondly, middlemen are an important and stable source for FBPG enterprises to purchase raw materials. At present, the government only provides a feed-in tariff subsidy for biomass power generation enterprises. If the enterprise transfers part of the subsidy to middlemen, the purchase quantity of middlemen will increase, and the profit of the enterprise will also increase. Therefore, enterprises can improve the supply enthusiasm of middlemen by means of increasing purchase price and ensure that the raw materials of FBPG enterprises meet the production capacity demand as much as possible. It also avoids the loss of stock shortage.

Finally, at the current stage, if the enterprise is expected to meet the production capacity demand, the purchase price of 425 yuan per ton is reasonable. In this case, the feed-in tariff can be increased to about 0.95 yuan per kWh to ensure the sustainable operation of biomass power generation enterprises. In addition, reducing the power generation operation cost of enterprises, promoting the use of brush cutters, reducing labor cost, and providing pruning subsidy can also promote the overall efficiency of the supply chain.

Although this paper simulates the reality of the FBPG supply chain in China as much as possible, there are still some details to be further considered due to the complexity of reality. For example, there is a time gap (usually one year) in the issuance of policy subsidy, which may lead to insufficient funds for enterprises to purchase biomass raw materials in that year, and many farmers think that it is difficult to prune, which may lead to a lack of labor. So middlemen need to hire labor from other provinces in China, increasing the cost of pruning.

These complex situations may become important factors hindering the development of biomass enterprises in China. Therefore, the prospects are put forward in the follow-up research:

1. The simulation model is only applicable to the forest biomass raw materials supply chain in the western region of China, which can be improved and optimized to make it applicable to other regions.
2. Continue to enrich the behavior rules of agents, such as the behavior rules of enterprises. The current setting of enterprise is that price is set on a uniform basis. As a result, farmers close to the enterprise can get rich income, while farmers far away can get less income. So the hierarchical pricing strategy can be further considered. There are different purchase prices for farmers at different distances, which can reduce the cost of enterprises.
3. The distribution of farmers, middlemen, and enterprise in the model is different from reality, so a regional map can be introduced to optimize the simulation effect.
4. Further discuss the problem of labor shortage in the western region of China.

## Figures and Tables

**Figure 1:** The supply chain system of FBPG.

**Figure 2:** Distribution of the woodland area.

**Figure 3:** Flowchart of farmer's behavior.

**Figure 4:** Flowchart of middleman's behavior.

**Figure 5:** Input parameters interface.

**Figure 6:** Main view interface.

**Figure 7:** Relationship between purchase price and purchase quantity.

**Figure 8:** Profit of the enterprise (price = 0.75).

**Figure 9:** Profit of the enterprise (price = 0.95).

**Figure 10:** The average profit of the agents of supply chain.

**Table 1:** Ways for farmers to sell raw materials.

Selling mode of farmers	Farmers sell to enterprises	Farmers sell to middlemen
Farmers take the initiative to transport	19	24
Farmers waiting to be acquired	4	7
Total	23	31

**Table 2:** Property and parameter setting of farmers.

Property	Letter representation	Meaning	Assigned value
Woodland area	FS	Woodland area owned by each farmer	141.06*e*^−0.523x^ mu

Farmer-enterprise distance	FEd	Distance from farmer to biomass enterprise	0∼300 km uniform distribution

Interval time of pruning	t	Time since last pruning	0∼5 years random distribution

Number of farmers	FNum	Number of farmers in the region	1000∼4000 (sliding strip)

Unit amount collected	UAmo	Quantity of raw materials collected per unit woodland	1 t/mu

Actual collection rate	*α*	Random factors such as season	0.5∼1 random distribution

Unit pruning cost	FCost	Cost of raw materials collected per unit woodland	70∼200 yuan/*t* (sliding strip)

Unit pruning subsidy	CSub	Government subsidy for unit woodland pruning	Input box input (yuan)

**Table 3:** Property and parameter setting of the middleman.

Property	Letter representation	Meaning	Assigned value
Middleman-enterprise distance	MEd	Distance from middleman to enterprise	100∼300 km uniform distribution

Number of middlemen	MNum	Number of middlemen in the region	10∼50 (sliding strip)

Middlemen purchase price	MPri	Price of raw materials purchased from farmer by middleman	150∼200 yuan (sliding strip)

Unit processing cost	MCost	Raw materials primary processing cost	20∼35 yuan/*t* (sliding strip)

**Table 4:** Property and parameter setting of the enterprise.

Property	Letter representation	Meaning	Assigned value
Enterprise purchase price	EPri	Purchase price of raw materials for enterprise	350 yuan/*t* (initial value)

Production capacity of the enterprise	EQua	Raw materials required for power generation when reaching production capacity	100000t

Unit power generation cost	ECost	Power generation cost of enterprise	0.292 yuan/kWh

Feed-in tariff	Price	Sale price per kWh	0.55∼1.55 yuan/kWh (sliding strip)

Purchase subsidy	GSub	Subsidy price of raw materials per cycle when production capacity is not reached	10 yuan/t

Raw materials conversion rate	*μ*	How much power is generated per ton of raw materials	800 kWh/t

**Table 5:** Type and performance of farmers' vehicles.

Vehicle type	Tricycle	Tractor	Four-wheel vehicle
Fuel consumption per 100 km (L)	10	15	20
Unit quantity of transportation (t/vehicle)	0.5	1.5	2.5

**Table 6:** Vehicle type and performance for middlemen.

Vehicle type	Large four-wheel vehicle	Truck
Fuel consumption per 100 km (L)	25	40
Unit quantity of transportation (t/vehicle)	5	30

**Table 7:** Profit index of agents under different purchase prices.

Profit index of agents	Epri = 380	Epri = 420
Number of farmers selling raw materials	331	411
Average profit of farmers	3930	4838
Number of middlemen	20	20
Average profit of middlemen	345867	435437
Number of enterprises	1	1
Average profit of enterprise	5264989	3586342
Total profit of supply chain	13483159	14283500

**Table 8:** Simulation experiment results of changing internal parameters.

Unit pruning cost (farmers)	The initial processing cost (middlemen)	Unit operating cost of power generation (enterprise)	Purchase price of enterprise when reaching production capacity	The feed-in tariff^*∗*^
100	25	0.292	420–430	0.95
70	25	0.292	285–295	0.65
100	20	0.292	420–430	0.95
100	25	0.25	420–430	0.70

^*∗*^The feed-in tariff here refers to the minimum price that can ensure that power generation enterprise does not suffer losses.

**Table 9:** Simulation experiment results of changing external parameters.

Number of farmers	Number of middlemen	Pruning subsidy	Purchase price of enterprise when reaching production capacity	The feed-in tariff^*∗*^
3369	20	0	420–430	0.95
3369	20	100	270–280	0.72
3000	20	0	515–520	1.05
3369	10	0	490–500	1.02

^*∗*^The feed-in tariff here refers to the minimum price that can ensure that power generation enterprise does not suffer losses.

## Data Availability

All data used in this paper are available from the authors upon request.
